The article "Influence of the enterprise’s intelligent performance evaluation model using neural network and genetic algorithm on the performance compensation of the merger and acquisition parties in the commitment period" was retracted in 2023. Reasons: unreliable results or conclusions; concerns about the peer review.

# Influence of the enterprise’s intelligent performance evaluation model using neural network and genetic algorithm on the performance compensation of the merger and acquisition parties in the commitment period

**DOI:** 10.1371/journal.pone.0248727

**Published:** 2021-03-19

**Authors:** Yuanyuan Luo, Da Ren

**Affiliations:** College of Management and Economy, Tianjing University, Tianjing City, China; Ministry of Natural Resources North Sea Bureau, CHINA

## Abstract

The purpose is to study the performance compensation of the bid purchased during the mergers and acquisitions (M&A) process. An intelligent model of enterprise performance appraisal is built to analyze the performances of the acquired enterprises. First, the evaluation indicators of enterprise performance are selected from both financial and non-financial aspects. An enterprise performance appraisal model is established based on the neural networks and optimized by the factor analysis method and Genetic Algorithm (GA). The principal factors affecting enterprise performance are analyzed. Then the M&A parties’ performances during the M&A commitment period under the earnings compensation mechanism are analyzed quantitatively. Corresponding hypotheses and evaluation indicators are established. Mean test results and regression analyses demonstrate that the hypotheses proposed are valid under particular circumstances. Introducing the earnings compensation mechanism during the M&A process can improve the enterprise performance effectively so that the earnings forecasted in the commitment period are significantly higher than the historical profitability. Hence, the earnings compensation mechanism plays a positive role in guiding enterprise performance. Comparison with models proposed in previous research reveals that the output error ratio of the designed corporate performance evaluation model is 1.16%, which can effectively evaluate corporate performance. The above results provide a reference for studying the impact of the earnings compensation mechanism on enterprise performance during the M&A process.

## 1. Introduction

The mergers and acquisitions (M&A) of an enterprise refers to its external expansion through equity transactions and capital operations, strengthening its development. As the economy boosts, industrial integration is accelerated, and the transaction scale of China’s M&A market increases significantly, with an increasingly tremendous quantity of large-scale M&A events. According to statistics, the total value of Chinese enterprises’ M&A in 2018 reached US$678.9 billion, an increase of 0.2% over 2017; the number of M&A transactions reached 10,887, an increase of 10.7% annually. In 2019, due to the decline in the number of global M&A, the volume and the number of transactions in China had decreased compared with 2018 [1]. In the M&A process, the asset pricing mechanism is the core, and the asset appraisal report in the M&A business is a vital basis for asset pricing, which can affect the success of an M&A project. Performance commitment refers to the commitment agreement signed by both M&A parties. During the commitment period, the acquired enterprise needs to make a commitment to its future performance to prove its value [2]. Signing an actual performance commitment can prevent M&A premiums and the inflated valuation of the acquired enterprise’s assets under the income approach. Therefore, it is indispensable to establish a reasonable and adequate enterprise M&A valuation model.

Ya et al. (2019) [3] studied the impact of M&A on the financial performance of listed enterprises. They investigated 434 M&A events initiated by Chinese listed enterprises in Shanghai Stock Exchange and Shenzhen Stock Exchange using data regression analysis. Results showed that value-chain-extension M&A and technology-seeking M&A were positively correlated to enterprise performance with other conditions unchanged. Enterprises could benefit from the operational scale in technology-seeking M&A, while the financial synergy brought by value-chain-extension M&A could improve enterprise performance [3]. Studying the influencing factors and indicator systems of enterprise performance worldwide, Yang et al. (2020) [4] established an indicator system for enterprise performance appraisal based on the two quantitative factors: financial performance and structure proportion. Then they used Artificial Neural Networks for adaptive training to obtain the optimized connection weights [4]. Sarraf and Nejad (2020) [5] ranked the importance of enterprise services through gray-level correlation analysis and obtained a reference sequence. Then they analyzed the data at all levels and measured the performance of the enterprise using the balanced scorecards [5]. Based on the balanced scorecard model combined with questionnaires, Zhao (2020) [6] constructed an enterprise performance appraisal model from the dimensions of finance, customers, internal processes, learning and growth, and environment. Then the backpropagation (BP) neural network and the Analytic Hierarchy Process were combined to determine the weight of each indicator, obtaining the actual appraisal model. The experimental results suggested that the balanced scorecard model helped improve an enterprise’s understanding of performance appraisal management. The neural network model could accurately predict the enterprise performance and provide sustainable development ideas for the enterprise [6].

Previous research suggests that the process of M&A will affect the overall performance of the enterprises, while the performance evaluation system can assess the performance of the enterprises. Therefore, an enterprise performance evaluation model is established based on the neural network model to study the performance compensation during the M&A commitment period. Moreover, the factor analysis and the genetic algorithm (GA) are innovatively introduced to optimize the results of the evaluation model, thereby improving the evaluation accuracy and computing power of the neural network model. Afterward, a profit compensation mechanism is introduced into the process of M&A, and the influence of the enterprise’s performance under this mechanism is analyzed. Relevant hypotheses and evaluation and analysis indicators are put forward, and the research problems are analyzed quantitatively. The research results can provide a reference for analyzing changes in the enterprises’ performance during M&A.

## 2. Method

### 2.1 Enterprise’s performance appraisal method based on BP-GA model

Enterprise performance appraisal uses statistical methods to comprehensively appraise the current performance and operating conditions of the enterprises based on a reasonable evaluation indicator system. With the increasing complexity of economic activities, enterprise performance appraisal can guide the innovation and development of enterprise management systems and enhance enterprise competitiveness [7]. The enterprise performance appraisal system comprehensively evaluates various factors affecting enterprise development according to different evaluation methods, rules, and data indicators. Usually, an enterprise performance appraisal indicator system is established based on financial indicators and non-financial indicators to accurately reflect the current operating conditions and future development capabilities of the enterprise. Financial indicators refer to the enterprise’s operational, financial analysis data, including indicators such as return on net assets, profit on the main business, and return on total assets [8]. Non-financial indicators include market share, customer satisfaction, research and development investment, and product quality, reflecting the innovation and development capabilities of the enterprise, as well as its future development [9].

Here, a sound performance appraisal indicator system is established to appraise enterprise performance comprehensively. An enterprise performance appraisal model is established based on the neural networks and optimized by the factor analysis method and GA. Finally, a comprehensive enterprise performance appraisal system is obtained. According to [10], appropriate evaluation indicators are selected from financial and non-financial aspects based on the research purposes, and a scientific and comprehensive performance evaluation system for enterprises is constructed, which can thoroughly evaluate the current production and operation status and the future development potential of the enterprises. The proposed performance evaluation indicator system is shown in Table 1.

**Table 1:** Enterprise’s performance evaluation indicator system.

Evaluation dimension	First-level indicator	Second-level indicator
Financial performance (A1)	Efficiency (B1)	Return on investment (C1)
		Return on net assets (C2)
	Development (B2)	The growth rate of net profit (C3)
		The growth rate of total assets (C4)
		Capital accumulation rate (C5)
		The growth rate of operating income (C6)
	Profitability (B3)	The turnover rate of accounts receivable (C7)
		Operating net profit margin (C8)
		Cost profit margin (C9)
		Return on assets (C10)
		Total asset turnover rate (C11)
		Inventory turnover rate (C12)
		Current assets to income ratio (C13)
		Basic earnings per share (C14)
	Solvency (B4)	Quick ratio (C15)
		Cash current debt ratio (C16)
		Current ratio (C17)
		Asset-liability ratio (C18)
	Cash (B5)	Cash content of operating income (C19)
		Net profit to cash ratio (C20)
	Risk (B6)	Financial leverage (C21)
		Operating leverage (C22)
Non-financial performance (A2)	Innovation (B7)	Research and development expenditure (C23)
		Number of patents (C24)
	Equity (B8)	The proportion of major shareholders (C25)
		The proportion of the top five shareholders (C26)

BP neural network has adaptive and self-learning capabilities. The output error of the network is reduced by assigning initial weights to the network, adjusting the output results of the network, comparing the output results with the expected value, and then adjusting the weights [11]. After many adjustment cycles, the output result of the network reaches the preset range, and the training of the network is completed. The BP neural network contains three layers: the input layer, the hidden layer, and the output layer. The three-layered network can apply to any nonlinear mapping and prevent the model from falling into local solutions due to excessive complexity [12]. The three-layered BP neural network designed here is shown in Fig 1.

**Fig 1:** A three-layered neural network.

The detailed algorithm flows are as follows [13]:

1. Appropriate input targets and data are chosen as sample data for training the network.
2. The network parameters are initialized, and a neural network model is established.
3. The sample data are utilized for training the network to reach the preset value cyclically.
4. The neural network is trained, its weight and threshold are obtained, and the result is output.

BP neural network’s algorithm flows are illustrated in Fig 2.

**Fig 2:** BP neural network’s algorithm flows.

Factor analysis belongs to Principal Component Analysis. It reduces dimensionality while preserving necessary information by mentioning public factors [14]. The constructed indicator system for enterprise performance appraisal includes 26 evaluation indicators. If these indicators are directly inputted into the BP neural network, the network structure will be too complicated. Hence, factor analysis is applied to process the enterprise performance appraisal indicators to improve the computing power of the neural network. Meanwhile, the high-dimensional data are transformed into multi-dimensional data, and the common factors in these data are extracted to obtain the significant connection between the indicators. The dimensionality of the neural network’s training samples is reduced to obtain eight comprehensive factors.

GA imitates the natural genetic processes, such as selection, reproduction, hybridization, and mutation. In each iteration process, a set of candidate solutions are retained, and the optimal solution is selected from individual groups according to the corresponding indicators. Therefore, a new generation of candidate solutions can be generated by repeating the biological, genetic processes, including selection, crossover, and mutation, until the indicators converge [15,16]. GA can obtain the best parameter settings through adaptive optimization search on parameters. The necessary steps of GA are explained as follows:

1. Coding: GA first requires coding operations to convert all candidate solutions in the problem into individuals that the algorithm can identify.
2. Generating the initial population: the entire algorithm is initialized by setting the initial population crossover range, mutation probability, and the number of population individuals.
3. Adaptation calculation: in the iterative process of the algorithm, each population individual needs to be evaluated and then sorted. The evaluation function used is the adaptation calculation. Different evaluation functions need to be defined for different problems.
4. Selection: individuals with good adaptation are selected as the next-generation population individuals (offspring) according to the fittest survival rule.
5. Crossover: some genes are exchanged for selected individuals with a particular probability, and crossover mode to produce new individuals based on the concept of population information exchange [17].
6. Mutation: various accidental factors in nature can cause individual genetic mutation. According to the individual evolution concept, the gene value of an individual is mutated with a particular probability so that the offspring produced has new characteristics that the parent did not have, and the diversity of the population is increased.
7. Calculation termination: when the generated offspring meets termination conditions, the individual with the most incredible adaptation in the new population is output as the optimal solution, and the calculation is terminated. If the individuals in the population do not meet the termination condition, the adaptation calculation process is continued until the termination condition is reached [18]. The calculation process is shown in Fig 3.

**Fig 3:** Calculation flows of GA.

GA only uses adaptation as the judgment criterion, without considering the continuity and differentiability of the problem and the expression of the objective function. Besides, it has excellent global searchability. The crossover and mutation operations can continuously generate new individuals, expand the search range of the optimal solution, obtain the optimal global solution through population evolution, and avoid falling into the local optimum [19].

In summary, according to the above analysis of the performance appraisal system, the BP neural network model is established and optimized by the factor analysis method and GA [20]. The specific process is:

1. The evaluation indicator data are selected, and the data dimensionality is reduced through the factor analysis method.
2. The parameters of GA are initialized, including population size and the maximum number of iterations.
3. The parameters of the BP neural network are initialized.
4. The reciprocal of each neural network layer’s output error square is taken as the adaptation function *VAL* of the value; the equation is:

$$VAL=\frac{1}{sumsqr(t-y)}$$ (1)

In (1), *t* represents the target value, and *y* represents the network output. The result of GA is used as the initial weight and threshold of the BP neural network.

(5) After the initial weight and threshold are obtained, the neural network begins training. After multiple iterations, the initial values and thresholds are updated until the desired effect is reached [21]. Then the training of the BP-GA model is completed. Finally, the BP-GA model based on factor analysis is obtained, and its algorithm flows are shown in Fig 4.

**Fig 4:** Algorithm flows of the factor analysis-based BP-GA model.

After the determined evaluation indicators are obtained, the required financial data are collected from the network platforms. First, the factor analysis method is adopted to evaluate the performance of the enterprise data; then, the results are input into the established BP-GA model, and the enterprise performance evaluation results are output.

### 2.2 Performance earnings compensation during the M&A process

Performance commitment refers to the commitment made by the acquired party to independently complete its performance within a period (usually 3 fiscal years) after the acquisition of the listed enterprise during the M&A process. The connotation of performance commitment is the amount of net profit attributable to the parent after the deduction of non-recurring losses after the upgrade. The purpose is to resolve the losses that the listed enterprise will ultimately bear due to the mismatch of information between the buyer and the seller during the M&A transaction [22]. Thanks to the basic national conditions in China, listed assets have a significant premium over non-listed assets, so that listed enterprises occupy a dominant position in the bargaining of purchases. Thus, the acquired party will undertake the commitment to complete the performance by rediscovering its value to become a part of the listed enterprise, eliminating the listed enterprise’s doubts about the value of the acquisition [23]. When a listed enterprise purchases the underlying asset, if the performance of the underlying asset reaches a threshold, the listed enterprise will pay an additional fee to the original asset owner as an adjustment to the original transaction consideration. This process is called valuation adjustment. Based on the cognitive differences in the value of the target in M&A transactions, the valuation adjustment gives the purchased party an opportunity to prove the value of the asset, which is a relatively fair clause [24]. Valuation adjustments belong to the price increase of listed enterprises, while price reductions are completed through compensation clauses for the inability of the purchased target to fulfill the performance commitment.

During the M&A process, to maintain the effectiveness of the M&A commitment, if the bid purchased fails to meet the performance commitment, it needs to compensate the listed enterprise. Generally, the compensation equation is:

CC=(CNI−ANI)×ACO÷CNI−CR (2)

In (2), *CC* represents the cash consideration that should be compensated for the *N*-th year, *CNI* represents the commitment to the total net profit of returnee deducted from non-recurrent loss in *N* years, *ANI* represents the actual total net profit of returnee deducted from non-recurrent loss in *N* years, *ACO* represents the consideration obtained from the original transaction, and *CR* indicates that the accumulated consideration has been compensated before [25]. In practice, both the compensation clause and the calculation method of the compensation consideration can be negotiated to reflect the risk characteristics and business characteristics of the industry in which the bid is purchased.

Compensation methods include cash compensation and equity compensation. Cash compensation requires the shareholders of the original bid purchased to pay cash to the listed enterprise. However, when the shareholders cannot provide so much cash, they will use the shares to compensate the listed enterprise through bottoming clauses [26]. In the way of equity compensation, the amount of consideration to be compensated needs to be divided by the unit price of the shares at the time of the M&A transaction to obtain the number of shares to be compensated. Then the listed enterprise repurchases the shareholders’ shares of the bid purchased at a price of 1 CNY before canceling the shares [27]. Shareholders of the original bid purchased who acquire the listed enterprise shares through the transaction must lock the enterprise shares they hold during the commitment period to avoid dumping the shares during the commitment period.

When the acquired party completes the performance commitment, it extracts part of the excess performance as a reward and distributes it to the team of bid purchased, which is called a performance bonus. The audience for valuation adjustments is the original shareholders of the bid purchased, focusing on verifying the judgments about the value of the bid purchased before and after the M&A [28]. In contrast, the audience for performance bonus is the core team of the bid purchased, focusing on encouraging the core team through incentives so that the team can create an excess performance for the listed enterprise and reduce the difficulty of integration after M&A.

Enterprise performance appraisal provides the feasibility for listed enterprises’ M&A, and the evaluation result of industrial assets determines the success or failure of listed enterprises’ M&A [29]. Enterprise performance appraisal is affected by various subjective and objective factors. To obtain more generous benefits, the acquired party will inevitably make the earnings forecast higher than historical profitability. Hence, the following hypotheses are made:

1. The earnings forecast of bid purchased are higher than historical profitability.
2. The earnings forecast of bid purchased are higher than actual profitability.
3. Earnings compensation mechanism can raise M&A valuation.
4. Earnings compensation will affect achieving earnings forecast targets.

Hence, the M&A earnings compensation is analyzed using the following indicators [30,31]:

1. *ER*_*t*_*dR*_*0*_: the ratio of the acquired party’s net profit *R*_*0*_ in the previous year before the M&A to the forecasted annual net profit during the commitment period *ER*_*t*_, calculated as:
  $$ER_{t}dR_{0}=\frac{R_{0}}{ER_{t}},\;t=1,2,3$$ (3)
2. *ER*_*t*_*dR*_*t*_: the ratio of the acquired party’s actual net profit during the commitment period *R*_*t*_ to the forecasted net profit of the current year *ER*_*t*_, calculated as:
  $$ER_{t}dR_{t}=\frac{R_{t}}{ER_{t}},\;t=1,2,3$$ (4)
3. *DevER*: the extent to which the total net profit forecast of the acquired party $\sum_{t=1}^{3}ER_{t}$ deviates from the actual total net profit $\sum_{t=1}^{3}R_{t}$, calculated as:
  $$DevER=\frac{\sum_{t=1}^{3}R_{t}}{\sum_{t=1}^{3}ER_{t}},\;t=1,2,3$$ (5)
4. *GroR*_*t*_: the annual growth rate of the acquired party’s actual net profit after the M&A, calculated as:
  $$GroR_{t}=\frac{R_{t}-R_{t-1}}{\left|R_{t-1}\right|},\;t=1,2,3$$ (6)
5. *AR*_*t*_*dR*_*0*_: the ratio of the net profit before the M&A to the average net profit during the commitment period ${\bar{R}}_{t}$, calculated as:
  $$AR_{t}dR_{0}=\frac{R_{0}}{{\bar{R}}_{t}}$$ (7)
6. The ratio of the net profit for one year after the expiration of the commitment period to the average net profit during the commitment period is:
  $$AR_{t}dR_{4}=\frac{R_{4}}{{\bar{R}}_{t}}$$ (8)
7. *PE*: the M&A price-to-earnings (PE) ratio represents the ratio of the purchase price BP to the average net profit predicted for the commitment period $\bar{E}{\bar{R}}_{t}$:
  $$PE=\frac{BP}{\bar{E}{\bar{R}}_{t}},\;t=1,2,3$$ (9)
8. M&A premium multiple refers to the ratio of the M&A bid’s purchasing price to the netbook asset *BV*:
  $$w=\frac{BP}{BV}$$ (10)
  The higher the M&A’s price-earnings ratio and premium multiple, the more challenging to achieve the committed forecast.
9. *ProImp* indicates whether the performance commitment is fulfilled. When *DevER* is <0, the performance commitment is not fulfilled, and *ProImp* is assigned a value of 0. When *DevER* is >0, the performance commitment is fulfilled, and *ProImp* is assigned a value of 1.
10. *VAM* indicates whether the earnings compensation mechanism is set during the M&A process. If the earnings compensation mechanism is not set, *VAM* is assigned a value of 0; if the earnings compensation mechanism is set, *VAM* is assigned a value of 1. *Stock* indicates whether equity compensation is adopted. If the equity compensation and cash compensation are adopted, *Stock* is assigned a value of 1; otherwise, it is assigned a value of 0.

One-sided T-test verifies and analyzes Hypothesis 1 and Hypothesis 2. A regression analysis model is constructed for empirical analysis of Hypothesis 3 and Hypothesis 4, and the equation is:

$$y_{i}=c+\alpha x_{i}+\varepsilon_{i}$$ (11)

In (11), *y*_*i*_ represents the explained variable, *x*_*i*_ represents the influencing factor variable, *α* represents the regression coefficient, *c* represents the constant term, and *ε*_*i*_ represents the random error term.

Here, the M&A case of an A-share listed enterprise in 2018 is taken as the research object. The data are screened to remove some imperfect data. Afterward, 203 sets of valid data that can verify Hypothesis 1 and Hypothesis 2 are obtained. A hundred and twenty-five sets of valid data that can verify Hypothesis 3 and Hypothesis 4 are obtained.

## 3. Results and discussion

### 3.1 Mean test analysis of Hypothesis 1 and Hypothesis 2

(1) Hypothesis 1: The earnings forecast of bid purchased is higher than historical profitability.

According to the results in Fig 5, the mean value of *ER*_*1*_*dR*_*0*_ is between 0.78–0.79. Except for the mean value of cash compensation, the mean values of other samples are significantly less than 1 at the 5% confidence level. The mean value of *ER*_*2*_*dR*_*0*_ is between 0.578–0.783, which is significantly less than 1 at the 1% confidence level. The mean value of *ER*_*3*_*dR*_*0*_ is 0.54–0.73, which is significantly less than 1 at the 1% confidence level. Therefore, the actual net profit of the three years after the M&A and the profit prediction is higher than the actual net profit of the year before the M&A. Moreover, the M&A stress prediction is significantly higher than the historical profit level. Therefore, Hypothesis 1 holds. In addition, the ratio of the net profit of the year before the M&A to the annual profit prediction after the M&A has decreased annually, indicating that the profit prediction for the first year after the M&A has increased significantly compared with the net profit of the previous year. Furthermore, earnings predictions are gradually shrinking from the previous year’s growth.

**Fig 5:** The empirical analysis of Hypothesis 1.

Hypothesis 2: The earnings forecast for bid purchased is higher than historical profitability.

Fig 6 suggests no mean value of profit compensation and cash compensation in *ER*_*1*_*dR*_*1*_, which is not significantly greater than 1 at the 5% confidence level. Moreover, there is no mean value of profit compensation in *ER*_*2*_*dR*_*2*_ and *ER*_*3*_*dR*_*3*_, which is not significantly greater than 1 at the 5% confidence level. Therefore, for the overall sample and the sample with profit compensation, the total value of the profit prediction for the three years after the M&A and the annual profit prediction are not higher than the actual profit level; thus, Hypothesis 2 does not hold. The total three-year stress prediction value of cash compensation and share compensation is lower than the actual profit. The value of share compensation can be predicted in the first two years, but cannot be predicted in the third year; the value of cash compensation cannot be predicted in the first year but can be predicted in the next two years. Therefore, under cash compensation, the pressure to achieve the profit prediction in the first year is greater; under the share compensation, the pressure to achieve the profit prediction is greater in the last year. Regarding the no-profit compensation, the total profit prediction for the three years after the M&A and the annual profit prediction are higher than the actual profit level. Hence, Hypothesis 2 is valid.

**Fig 6:** The empirical analysis of Hypothesis 2.

### 3.2 Regression analysis of Hypothesis 3 and Hypothesis 4

Hypothesis 3: Earnings compensation mechanism can raise M&A valuation.

Hypothesis 4: Earnings compensation will affect achieving earnings forecast targets.

According to the results of regression analyses presented in Figs 7 and 8, *VAM* and Stock have significant impacts on enterprise performance, indicating that introducing an earnings compensation mechanism will affect M&A valuation. However, equity compensation cannot impact M&A valuation significantly. Therefore, Hypothesis 3 holds. Introducing the earnings compensation mechanism and adopting the earnings compensation method of equity compensation will affect the fulfillment of the target earnings forecast. Hence, Hypothesis 4 is valid.

**Fig 7:** The empirical analysis of Hypothesis 3.

**Fig 8:** The empirical analysis of Hypothesis 4.

### 3.3 Model verification

The data of a product supplier are selected, processed after normalization, and input into the Bayesian network model [32], average support vector machine (ASVM) model [33], BP neural network model [34], PSO-BP neural network, RBF neural network model [35] and the designed and trained BP-GA model to test the evaluation results of the proposed model on enterprise performance and prove the effectiveness and feasibility of its application. The simulation test is based on factor analysis. The comparison between the output result of the model and the expected result is shown in Fig 9.

**Fig 9:** Results of model verification.

As shown in Fig 9, different models have different evaluation results on enterprise performance. Among them, the Bayesian network-based performance evaluation model has the largest output error ratio of 3.88%; the BP-GA model has the smallest output error ratio of 1.16%. Therefore, compared with the algorithms proposed in previous studies, the BP-GA model based on factor analysis can effectively evaluate enterprise performance.

In summary, the profit prediction and performance compensation under the profitability of M&A are researched, and the cases of M&A are analyzed by constructing empirical analysis indicators. The mean test and regression analysis methods are combined to verify the hypotheses. Results suggest that in the process of M&A, the stress prediction value of the M&A target in the commitment period is higher than the historical profit level. Under the condition of profit compensation, the deviation from the historical profit level will be higher than that of no profit compensation. Introducing a stress compensation mechanism will positively affect the performance of the target enterprise during the commitment period, which will lead to earnings management behavior before M&A. Besides, the proposed model is compared with performance evaluation models of previous studies. The results show that the designed BP-GA model based on factor analysis has a lower output error ratio (1.16%), which can effectively evaluate the performance of the enterprise before and after the M&A.

## 4. Conclusion

An enterprise performance evaluation indicator system is established to study the performance compensation of both parties in the M&A process. Then an enterprise performance evaluation model is established based on BP neural network and optimized by factor analysis and genetic algorithm for intelligent analysis of enterprise performance. Afterward, the performance commitments of both parties in the M&A are analyzed. The profitability of the M&A is selected for discussion, and relevant hypotheses and evaluation indicators are put forward. The experimental results demonstrate that in the process of M&A, the profit compensation mechanism will improve the enterprise performance, obtain a higher stress prediction value than the historical profit level, and bring positive guidance to the enterprise performance. Compared with the models in previous research, the output error ratio of the designed performance evaluation model is 1.16%, which is better than the output results of other models. Thus, it can effectively evaluate enterprise performance. However, there are several shortcomings found. The M&A process is finished by the agreement and system associated with customs clearance. Therefore, it is difficult to measure and analyze the relevance of the events. Hence, more complex measurement models will be adopted in the following research.

## Supporting information

S1 Data (ZIP)
